The article "Study on the Impact of Chinese Comedy International Communication on the Health of Older People under Cultural Ecological Environment" was retracted in 2023. Reason: compromised peer review.

# Study on the Impact of Chinese Comedy International Communication on the Health of Older People under Cultural Ecological Environment

**DOI:** 10.1155/2022/4003853

**Published:** 2022-07-12

**Authors:** Yan Zhang, Wang Wu, Jie Wei

**Affiliations:** ^1^School of Management, Guangzhou College of Technology and Business, Guangzhou 510580, Guangdong, China; ^2^Logistics Management, Wuhan Business School, Wuhan 430056, China; ^3^Electronic Information Science and Technology, Jiangsu Ocean University, Lianyungang 222005, Jiangsu, China

## Abstract

There are many kinds of works in Chinese comedy culture, which are deeply loved by audiences at home and abroad. In order to explore the impact of the international spread of Chinese comedy culture in the ecological environment on the health of the elderly public, this study studied these elderly comedy audiences from the aspects of age, monthly income, physical health, mental health, and public stability through statistical methods. The results show that the international spread of Chinese comedy culture is conducive to the physical and mental health of the elderly public, relieves the pressure of life, and ultimately contributes to social harmony and stability.

## 1. Introduction

The types of works in China's comedy culture market are divided into film and television comedy, stage comedy, and humorous quyi. In addition to traditional humorous quyi, such as cross-talk and storytelling, talk shows, and sketches in quyi, stage drama comedy and film and television comedy belong to the form of comedy combining Chinese and Western. Film and television comedies with low threshold and stage comedies and humorous quyi with high consumption form cultural products for healthy consumption of consumers at different levels. And because of the mobile phone short video and other auxiliary communication tools, humorous quyi and stage comedy, which usually consume thousands of yuan to thousands of yuan, can also realize people-friendly communication, forming a unique comedy form such as hilarious online segment video. When watching comedy culture, consumers of different ages and monthly incomes can mediate their mood, relieve their inner emotions, and let the elderly audience relax, so as to promote social harmony and stability. Comedy cultural products can make the audience fully relax and alleviate the pressure of life, so as to achieve the ultimate goal of promoting public health. With the development of China's comedy culture market, we should increase the breadth and depth of the content of comedy culture, improve the original effect of comedy itself, pay more attention to the objectivity and effectiveness of supervision and audit, and let China's comedy culture play a greater positive role in the process of international communication in the ecological environment because laughter can not only meet other human needs but also meet other human needs at more levels. At the same time, comedy laughter can also meet the needs of human beings at all levels. Psychological balance can make people calmly deal with the changing environment around them, so as to achieve health and longevity. In real life, not all goals can be achieved and all needs can be met. Setbacks and failures are inevitable. Anxiety and tension will often invade the body and mind. In the ecological environment, the spread of Chinese comedy culture can relieve tension and anxiety while relaxing and enjoying. It helps to eliminate physical and mental fatigue and maintain immune mechanism, improve life vitality, and strengthen physical strength and energy.

This study used statistical methods to deeply study the impact of Chinese comedy on the elderly public health, mainly through the audience analysis of consumers of different ages and different monthly incomes on different cultural communication platforms and comedy culture in terms of physical health, mental health, and public stability. The results show that comedy culture is conducive to the physical and mental health development of the audience; the previous cultural communication methods and comedy culture can no longer meet the needs and development of the public. Today, with the high development of science and technology, it provides new ideas, new methods, and new platforms for the communication of Chinese comedy culture. Knowing that the improvement of living standards and the pressure of life make the spiritual needs of the elderly public more and more intense and relieve the pressure of depression and anxiety, we can help alleviate our inner emotions through the appreciation of comedy culture, so as to ensure the health of the elderly public.

## 2. Literature Review

Liu, due to the rapid development of domestic comedy films, can bring spiritual enjoyment to the audience. At the same time, the entertainment consumption market of cinemas is also increasing day by day and has made good achievements. The spiritual needs of consumers are also higher and higher, which can make the audience feel happy in the comedy culture [1]. Xie and Chang described that comedy aesthetic education is related to the shaping of the national soul and the spiritual construction of the times. Therefore, strengthening the role of the wind vane of the mainstream media, increasing the demonstration and guidance of high-quality comedies, strengthening the education of comedy aesthetics in schools, and building and optimizing the three-dimensional system of comedy communication are the only way to build a harmonious and healthy comedy aesthetics and can promote the dissemination and development of Chinese comedy culture [2]. In recent years, comedy plays a more and more important role in China's entertainment consumer market, and the audience's demand for comedy is becoming stronger and stronger. Wang takes the traditional comedy culture company as the main research object. By analyzing the strategic decision of its commercialization transformation, he summarizes the correct direction and value orientation of the comedy culture industry chain and then explores the comedy industry marketing strategy with both innovation and general moderation [3]. Li and Wu under the changes of the times, the comic spirit has become an important feature in his creation, giving new aesthetic symbols to contemporary literary creation. This paper expounds the connotation of comic spirit and discusses the gradual change of comic spirit in literature since the new era [4]. Liu as relaxed, humorous, sharp, and interesting literary and artistic content has become the rigid demand of the current society; comedy culture has begun to penetrate into all aspects of literary and artistic creation and also reflects the changing aesthetic trend of the times [5]. Hao in recent years, the application of short video, has grown rapidly. Its communication mode of integrating video, listening, sound, and painting has updated the habits of modern people to receive information and socialize. At the same time, it also provides a new platform for knowledge communication, such as traditional culture communication, and has attracted the attention of a large number of audiences [6]. The material of comedy comes from life. The good things and memories in life are worth recording, so as to awaken the love of comedy culture. With the development of comedy, it can be seen that comedy can bring more and more happiness to the public, whether it is physical or psychological. Zang based on comedy culture, starting from the psychology of the audience and through the localized creative mode, rendered the atmosphere of empathy, so as to realize group empathy and continue the spiritual core of comedy; and cater to the aesthetic preference of the audience in the consumption era. Emotionally, it carries the space of empathy, soothes the inner dilemma and anxiety of modern people through emotional resonance, and better promotes public health [7]. Xie and Cheng pointed out that comedy culture must break through the international siege and explore and tap the comedy phenomenon and comedy spirit in real life in the comedy consciousness [2].

## 3. Analysis of Chinese Comedy Audience

With the development of Chinese comedy culture, there are many types of comedy, such as comedy film, comedy theater, and music comedy.  Table 1 provides the viewing platforms of comedy audiences according to different ages and the number and proportion of each type of comedy audience.

In Table 1, comedy audiences younger than 25 years old tend to watch comedies in cinemas and through mobile phones when they watch comedies through cinemas, grand theaters, small stages in bars, computers/tablets and mobile phones, which is easier for contemporary young people to reach; comedy audiences aged 25–35 prefer to watch comedy through mobile phones and small stages in bars; audiences aged 35–50, like comedy audiences aged 25–35, watch comedy mainly through mobile phones and small stages in bars; when they are older than 50, they mainly watch comedies through mobile phones and bars.  Figure 1 is drawn following the data in Table 1 to facilitate readers' understanding and comparison of the data.

As shown in Figure 2, the audience for comedy in the cinema decreases with age, that is, most of the people who go to the cinema are young people, and the older audience rarely goes to the cinema to watch comedy programs, but through mobile phones, computers, or tablets; on the contrary, the audience who watch comedy through the small stage of the bar increases with age [8].

At the same time, the monthly income of these comedy audiences is grouped to see the impact of different consumption levels on these audiences. After statistics, the data in Table 2 are obtained.

In Table 2, it can be seen from the data that comedy audiences with a monthly income of less than 3000 watch comedy mainly through mobile phones, computers, tablets, and cinemas, which do not need consumption or have low consumption. With the increase of income, it is not limited by this. You can watch comedy in theaters or bars. Figure 2 is drawn based on the data in Table 2 to facilitate a better understanding of the data.

In Figure 2, when the income is more than 8500 yuan, all ways to enjoy comedy are evenly distributed, about 20%. Most audiences at this income level have no consumption restrictions and can enjoy comedy at will. With the decrease in monthly income, the proportion of watching through mobile phones increases.

## 4. The Influence of Comedy Appreciation on Residents' Mental Health

To study the impact of watching comedy on the mental health of the elderly audience, the depression and anxiety of the elderly audience were rated. The data in Table 3 were obtained by classifying the length of time of enjoying comedy.

In Table 3, it can be seen that the score of depression and anxiety rating for the audience who did not enjoy comedy is higher, while the score of rating decreases with the increase of the time of enjoying comedy, but the score will increase after the time is longer than 4 hours, which also shows that not watching comedy for a long time will also affect people's mental health and make people anxious.  Figure 3 is drawn following the data in Table 3.

It can be seen from Figure 3 that the rating scores of depression and anxiety develop in a U-shape with the increase of time, which shows that there is an optimal time for watching and appreciating comedy, rather than the longer the time, the better. Beyond the best time, appreciation time is not conducive to the mental health development of the elderly audience.

## 5. Impact of Comedy Appreciation on Residents' Physical Health

After analyzing the mental health of the elderly audience who appreciate comedy, we will make a statistical analysis on the physical health of the elderly audience and make statistics on the prevalence of various diseases of the elderly audience watching for different lengths of time, so as to obtain the data in Table 4.

In Table 4, it can be seen from the data of various physiological diseases that the appreciation of comedy can reduce the prevalence of diseases such as three high and ventilation, which shows that watching comedy programs can adjust the physical function of the elderly, which is conducive to the healthy development of the elderly.  Figure 4 is drawn based on the data in Table 4.

It can be seen from Figure 4 that with the extension of comedy appreciation time, the probability of suffering from various diseases will be reduced, which shows that comedy appreciation can be used to maintain the health of the elderly audience.

## 6. The Role of Comedy in Maintaining Stability of the Chinese Public

This study mainly discusses the impact of the international spread of Chinese comedy culture on the elderly public health. The above research is from the aspects of physical health and mental health and then from the aspect of social public stability maintenance, mainly from four observation indicators. The data are statistically analyzed to obtain the data in Table 5.

In Table 5, it can be seen that the audience who did not watch comedy scored higher on social contradictions and social negative factors, and the score will gradually decrease with the increase of the duration of enjoying comedy.  Figure 5 is drawn following the data in Table 5.

As shown in Figure 5, the longer you watch comedy, the lower your score on social contradictions and social negative factors, which shows that watching and appreciating comedy is beneficial to the people with social contradictions and negative attitudes, the physical and mental health of the elderly audience, and the stability of the public.

## 7. The Overall Development View of Chinese Comedy

### 7.1. Appropriately Increase the Channels for the Masses to Contact International Chinese Comedies

With the further development of China's economy, the number of screens in China shows a high growth trend. At the same time, the income of Chinese people begins to enter the level of middle-income countries, and most people have entered a well-off life. However, it also faces a series of problems, such as difficult medical treatment, expensive school, serious social polarization between the rich and the poor, environmental pollution and so on. Many ordinary people will feel the depression and helplessness of life. At this time, they will find a way to relieve their worries and vent their emotions. Therefore, there are more and more comedies, and the market is getting hotter and hotter. Comedies spread and develop rapidly in various ways. The audience of online self-made sitcoms is mainly young people. They watch online self-made sitcoms with entertainment, catharsis, curiosity hunting, and conformity. At the same time, two-way and multidirectional communication interaction has been formed between the audience, video websites, and the audience. Nowadays, there are more and more elderly people, and the lineup of the elderly audience is also larger and larger. Pay attention to the concerns of the elderly audience, from scientific health preservation to promising old people, and enrich the spiritual life of the elderly.

In Zhu's analysis of the program innovation of “happy comedian” from the perspective of communication, taking “happy comedian” as an example, the hit volume in TV stations and online videos reached more than 10 billion. Through the integration of cross-talk, sketch, juggling, quyi, mime, and other forms, it improved the cultural connotation of the program, expanded the program communication channels, enriched the audience integration mode, and created a unique cultural communication direction of comedy variety shows [9]. Wang and Wang mentioned in their discussion on the emergence and characteristics of online dramas that online comedies have grown from scratch, from self-made online dramas to phenomenal popular online dramas, and then to the more diversified content of online comedies. The audience has also changed from one-way recipients to users who can choose and participate, with changes in attitude and action [10]. Qian in the positive role of comedy short video in the dissemination of urban image, taking comedy short video as an example, in the Internet era, various short video software are rising rapidly. Short video has strong communication function and commercial value, and its integration degree is high [11]. Rao and Yin mentioned in the new pattern of Chinese films and comedy film creation that the increase of hardware facilities of domestic comedy films, such as the number of screens in cinemas and the growth of new communication channels, has also increased the capacity of the market [12]. Under the macro background of the country's vigorous development of creative industry, the communication mode of contemporary Chinese comedy has long been derived from a single stage to a broader media platform. The centralized outbreak of Chinese comedy is also the result of the joint action of internal and external factors of Chinese films. The pressure in life makes more people choose comedy culture to alleviate their inner emotions, feel comedy culture through different communication platforms, better develop comedy channels, and further promote the development of comedy culture. The diversity of comedy development makes the acceptance of comedy by the elderly audience more and more common. The value judgment in comedy culture will also make the elderly audience aftertaste the value of comedy culture after laughing.

### 7.2. Properly Control the Social Phenomenon of Excessive Consumption

From the current development of China's comedy market, some works are over marketed, the content is single, ignoring the commitment of social responsibility, lack of guidance to teenagers, lack of thinking about the real society, and ignore the bottom line of moral principles. Both the form of expression and the content of the story have lost their cultural value. In particular, some low-cost comedy films blindly imitate and follow the trend in order to achieve high box office. Although the content of the works is humorous, they have lost the cultural value of comedy itself. Chinese comedy has achieved diversified development in the form of creation, and its strong local advantages have become an effective weapon for the differentiated competition between Chinese films and foreign commercial films. But there are also many problems behind the wonderful, such as the narration, creativity and branding of Chinese comedy films. We must further improve the quality and win the audience and market in order to win the space for sustainable development. Chinese comedies seem to be trying their best to get rid of the image of “vulgar.” In addition to the funny bifurcated passages, whether the works can bring emotional resonance to the audience is successful. The performance form of comedy culture is characterized by illogical and slightly neurotic. The colorful performance form and vulgar comedy culture will make the audience laugh happily. After that, it has no value of comedy connotation. It needs to arouse deep thinking. When winning the box office, we should also pay attention to the dissemination of the value of comedy culture. Chinese comedy is an indispensable part of domestic films, and the audience's demand for Chinese comedy films is also higher and higher. Generally speaking, in the future development of Chinese comedy, we should deal with these problems in time; otherwise, it will lead to the audience's aesthetic fatigue of Chinese comedy, thus losing attention, and the decline of Chinese comedy is not far away.

### 7.3. Develop New Forms of Comedy with Local Cultural Centers as the Core Force

Cultural centers are institutions that carry out mass cultural activities and provide places for cultural and recreational activities. With people's higher and higher requirements for cultural level and various types of activities emerging one after another, cultural centers in various regions have added relative measures to improve grass-roots culture. To improve the cultural heritage and quality of the people, infiltrate culture into people's daily life and let high-quality culture enter people's life. The cultural center takes a people-oriented position and starts from different aspects to meet the cultural and artistic needs of the public. The popularization of culture and art has become the central task of the new era cultural center, in which comedy culture has become a hot spot. In recent years, new comedies have appeared around the public in various forms. To effectively popularize and promote new comedies, present comedy culture to the public with a high-quality appearance, and make the new comedy cause develop more standardized and healthy, various activities can be organized with the help of the operation and venue of the cultural center, carry out promotion and training in local cultural centers, go deep into the grass-roots people, listen to their ideas and opinions, summarize and standardize their opinions, fully meet the needs of the people from literary and artistic creation, public welfare training, group cultural activities, free opening and other service programs, and develop new comedies with local cultural centers as the core force, which not only shows the people's demand for comedy culture but also shows the state's support for comedy culture, The integration of advantages between comedy cultural centers can enhance exchanges between the masses, so that the people with comedy talent and interested in comedy can actively participate in it, so that they have a platform to learn and show themselves, so that their way of humor can be transformed into a force to pass happiness to more people.

## 8. Conclusion

Based on the international communication of Chinese comedy culture, this study studied the impact on social public health. Through statistical methods, this paper analyzes and compares the aspects of different ages, different monthly incomes, physical health, mental health, and public stability and comes to the conclusion that comedy culture is conducive to the physical and mental health of the elderly audience and the stability of the public. The development of the Chinese comedy culture market under the ecological environment has a certain influence on the international communication of comedy culture. Therefore, it is necessary to expand the path of comedy culture communication and better promote the international communication of Chinese comedy.

## Figures and Tables

**Figure 1:** Audience analysis of Chinese comedy under the age group.

**Figure 2:** Analysis of Chinese comedy audience under the income group in February.

**Figure 3:** Analysis of the impact of comedy appreciation on residents' mental health.

**Figure 4:** Analysis of the impact of comedy appreciation on residents' physical health.

**Figure 5:** Analysis of the role of comedy in maintaining stability of the Chinese public.

**Table 1:** Audience analysis of Chinese comedy by the age group.

Grouping	<25	25–35	35–50	>50
Cinema	22.9	14.2	5.3	3.6
Grand theater	7.8	11.3	11.5	6.9
Bar stage	15.4	18.3	25.5	33.6
PC/tablet	8.6	14.1	19.1	22.4
Mobile phone	45.3	42.1	38.6	33.5

**Table 2:** Audience analysis of Chinese comedy by the income group in February.

Grouping	<3000	3000–5500	5500–8500	>8500
Cinema	18.2	22.4	23.1	19.6
Grand theater	3.3	7.8	10.9	15.6
Bar stage	12.7	19.2	21.5	22.4
PC/tablet	20.6	18.3	19.2	20.8
Mobile phone	45.2	32.3	25.3	21.6

**Table 3:** Impact of comedy appreciation on residents' mental health.

Grouping	0 h	1 h	2 h	3 h	4 h	5 h
Depression rating	6.39	5.29	5.08	4.92	4.96	5.36
Anxiety rating	6.18	5.03	4.85	4.73	4.81	5.16

**Table 4:** Impact of comedy appreciation on residents' physical health.

Grouping	0 h	1 h	2 h	3 h	4 h	5 h
Three high	21.6	19.3	18.6	18.1	17.9	17.8
Improve air circulation	5.2	4.9	4.7	4.6	4.5	4.5
Gynaecopathia	24.3	22.5	21.4	20.6	20.3	20.1
Andrology	18.6	17.1	16.3	15.8	15.6	15.5
Endocrine disorder	32.4	30.9	28.7	28.1	27.8	27.6

**Table 5:** The role of comedy in maintaining the stability of the Chinese public.

Grouping	0 h	1 h	2 h	3 h	4 h	5 h
Family contradiction	27.6	24.3	23.5	23.1	22.7	22.4
Contradiction between cadres and the masses	18.2	16.3	15.9	15.7	15.6	15.5
Make trouble	4.9	4.2	3.9	3.7	3.6	3.5
Campus violence	8.7	7.2	6.8	6.5	6.4	6.4

## Data Availability

The data used to support the results of this study are included within the article.
